# Assessing the Mechanism of Action of “Fructus Ligustri Lucidi-Cuscutae Semen” in Prostate Cancer Treatment Using Network Pharmacology and Molecular Docking

**DOI:** 10.1155/2022/7543619

**Published:** 2022-10-25

**Authors:** Dongdong Lu, Jianwei Shang, Xiping Guo, Yaosheng Zhang

**Affiliations:** ^1^Graduate School of Beijing University of Chinese Medicine, China; ^2^Department of Andrology, Dongzhimen Hospital, Beijing University of Chinese Medicine, China

## Abstract

**Objective:**

To explore the mechanism of action of “Fructus Ligustri Lucidi-Cuscutae Semen” in the treatment of prostate cancer using network pharmacology and molecular docking.

**Methods:**

The active ingredients and targets of “Fructus Ligustri Lucidi-Cuscutae Semen” were obtained by searching the TCMSP and DrugBank databases. These were matched and corrected using the UniProt platform. A drug “active ingredient-target” network map was constructed using Cytoscape 3.8.0. Prostate cancer-related targets were acquired from GeneCards, Disgenet, DrugBank, and other databases. The protein-protein interaction (PPI) network between the drug and prostate cancer was constructed with BioGenet; the crossover network of the two targets was extracted derive the key targets of “Fructus Ligustri Lucidi-Cuscutae Semen” for prostate cancer treatment. We used the Metascape platform for GO and KEGG enrichment analysis of the key targets. AutoDockTools1.5.6 and PyMOL software were used to perform molecular docking.

**Results:**

We obtained 13 active ingredients, 221 drug targets, 1511 prostate cancer targets (including 221 key targets), and 305 KEGG pathways from “Fructus Ligustri Lucidi-Cuscutae Semen.” Paclitaxel, quercetin, kaempferol, TP53, *β*-sitosterol, EGFR, and ESR1 in “Fructus Ligustri Lucidi-Cuscutae Semen” showed good docking activity.

**Conclusion:**

“Fructus Ligustri Lucidi-Cuscutae Semen” is a valuable clinical guide for the treatment of prostate cancer with multicomponent, multitarget, and multipathway characteristics.

## 1. Introduction

Prostate cancer (PCa) is a common disease of the male urinary system that causes malignant tumours in men. It has high incidence and mortality [1]. PCa treatment consists of hormones, radiotherapy, and surgery [2]; however, its side effects and complications cannot be ignored. By contrast, Chinese medicine has significant adjuvant treatment prospects for PCa that can effectively alleviate the side effects and complications, prolong the survival of patients, and reduce tumours.

Fructus Ligustri Lucidi and Cuscutae Semen are traditional Chinese herbs that are commonly recommended for the treatment of patients with advanced tumours. These plants have antitumour and immune function enhancing effects; however, the underlying mechanisms of action involved in the treatment of prostate cancer have not been fully elucidated [3].

The application of network pharmacology to construct a “drug-compound-target-disease” network for multidirectional pathway research makes the material basis and mechanism of action of herbal medicines and compounds more systematic. This can compensate for the limitations of single pathway research into herbal medicines and develop an understanding of the holistic and multidirectional nature of herbal medicines in treating diseases [4, 5]. “Drug-disease” target prediction is beneficial to guide scientific research ideas and the development of new tumour drugs. In this study, we analysed the potential active ingredients and targets of “Fructus Ligustri Lucidi-Cuscutae Semen” through network pharmacology. Additionally, we explored the molecular biological mechanism of its treatment in PCa to provide guidance for future basic research and combined Chinese and Western medicine treatments.

## 2. Materials and Methods

### 2.1. Active Ingredients and Target Prediction of “Fructus Ligustri Lucidi-Cuscutae Semen”

The TCMSP database (https://old.tcmsp-e.com/tcmsp.php) was searched for all the active ingredients of Fructus Ligustri Lucidi and Cuscutae Semen. These were integrated, and any duplications were removed. Any components that passed the ADME screening criteria of oral bioavailability (OB) ≥ 30% and drug-likeness (DL) ≥ 0.18 [6] were imported into the TCMSP platform to obtain the targets from the DrugBank database. The validated targets with the species “Homo sapiens” were screened and imported into the Uniprot database (https://www.uniprot.org) and standardised to the officially recognised gene names.

### 2.2. Construction of the “Active Ingredient-Target” Network of “Fructus Ligustri Lucidi-Cuscutae Semen”

Cytoscape 3.8.0 software was used to build and analyse the “active ingredient-target” network diagrams of “Fructus Ligustri Lucidi-Cuscutae Semen.” The “node” and “edge” represented the ingredient or target and the relationship between them, respectively. The network parameters, such as degree, betweenness, and closeness, were analysed using the Network Analyzer plug-in in Cytoscape 3.8.0. By analysing these network parameters, the key active ingredients, targets, and their relationships in “Fructus Ligustri Lucidi-Cuscutae Semen” were investigated.

### 2.3. Prostate Cancer-Related Target Search

We explored GeneCards (https://www.genecards.org/), OMIM (https://omim.org/), and Disgenet (https://www.disgenet.org/) for potential targets for the treatment of PCa using “prostate cancer” as a keyword. In the GeneCards database, targets were screened with a relevance score > 10. The results of the three databases were pooled, and duplicates were removed to obtain the final disease targets for PCa.

### 2.4. PPI Network Construction and Key Target Screening

Protein-protein interaction (PPI) networks were completed using BisoGenet. The active ingredient targets of Fructus Ligustri Lucidi and Cuscutae Semen, and PCa targets, were successively entered into BisoGenet to generate a PPI network. The intersection of the two PPI networks was extracted using the Merge plug-in within Cytoscape 3.8.0. This extracted the intersection network of the two PPI networks and analysed the properties of each node in the intersection network using CytoNCA [7]. Next, the median of connectivity, *k*1, was calculated; all nodes with connectivity >2 × *k*1 were selected, i.e., “Hit hubs.” The properties of each node in the Hit hubs network were calculated to obtain the degree centrality (DC), closeness centrality (CC), and betweenness centrality (BC). The core targets were selected based on the properties of all nodes.

### 2.5. Pass-Through Enrichment Analysis

The enrichment analyses commonly used in network pharmacology are GO functional enrichment analysis and KEGG pathway enrichment analysis. The main function of GO analysis is to predict the relationship of potential targets in terms of biological process (BP), molecular function (MF), and cell composition (CC). KEGG analysis maps these molecular objects or targets to molecular interaction, reaction, or relation networks. Potential targets were entered into the Metascape database (https://metascape.org/) for the GO and KEGG analysis. Data were visualised using Image GP (http://www.ehbio.com/ImageGP/).

### 2.6. Molecular Docking

To verify the reliability of the key targets of “Fructus Ligustri Lucidi-Cuscutae Semen” in the treatment of PCa, we performed molecular docking between the potential active ingredient and key targets. The 3D structures of the key target proteins (resolution, <2A) were obtained from the PDB database (https://www.rcsb.org). The 3D structures of the active ingredients were obtained through the PubChem platform. PyMOL was applied to remove ligands and water molecules. AutoDockTools 1.5.6 was used to hydrogenate the target proteins, calculate the charge number, and determine the AD4 type of the atoms. The built-in plug-ins, autogrid4 and autodock4, were run to determine the binding energy of the best docking site between the active ingredient and target protein. Finally, PyMOL was used to draw a molecular docking map and derive the docking hydrogen bond distance and docking target name for optimization and output.

## 3. Results

### 3.1. Active Ingredients and Target Acquisition of Fructus Ligustri Lucidi and Cuscutae Semen

In this study, 148 active ingredients of Fructus Ligustri Lucidi and Cuscutae Semen were obtained by searching the TCMSP database; eight active ingredients of Fructus Ligustri Lucidi and eight active ingredients of Cuscutae Semen were screened using the OB ≥ 30% and DL ≥ 0.18 criteria. Of these, three active ingredients overlapped between the two (active ingredients are listed in Table 1). The TCMSP database yielded 194 and 204 targets for Fructus Ligustri Lucidi and Cuscutae Semen, respectively, from the DrugBank database. The UniProt database was used to convert protein names to gene names.

### 3.2. Construction and Analysis of the “Active Ingredient-Target” Network of “Fructus Ligustri Lucidi-Cuscutae Semen”

The relationship network of potential active ingredients and targets of action of Fructus Ligustri Lucidi and Cuscutae Semen was obtained using Cytoscape 3.8.0. The network analyzer plug-in analysed topological parameters to assess the importance of the active ingredients and targets of action. In total, 234 nodes (containing 221 targets and 13 active ingredients) with 414 relationships were obtained (Figure 1).

### 3.3. PCa-Related Target Search

As of January 2022, the GeneCards, OMIM, and Disgenet disease databases were searched using the keyword “prostate cancer.” In the GeneCards, we exported data in Microsoft Excel format and set the relevance score to >10 to filter for potential targets for PCa; 1453 potential targets were obtained. The OMIM-entry-retrieval file was downloaded directly from the OMIM database; 156 potential PCa targets were obtained after screening and deweighting. In the Disgenet disease database, 209 potential PCa targets were obtained after screening and deduplication. After aggregating the above targets and removing any duplicates, the final number of potential PCa targets was 1511. The 221 drug targets and 1511 disease targets were imported into Venny 2.1 to obtain 132 common targets. The intersection of the two Venn diagrams is shown in Figure 2.

### 3.4. PPI Network Construction and Key Target Screening of “Fructus Ligustri Lucidi-Cuscutae Semen” for the Treatment of PCa

#### 3.4.1. PPI Network Construction of “Fructus Ligustri Lucidi-Cuscutae Semen” for the Treatment of PCa

The PPI networks of “Fructus Ligustri Lucidi-Cuscutae Semen” and PCa were constructed by using the BisoGenet plug-in in Cytoscape 3.8.0. There were 7703 targets directly or indirectly interacting with PCa and 173861 relationships between these targets. Moreover, there are 12435 targets directly or indirectly related to PCa and 239731 relationships between these targets. The intersection network between the two is shown in Figure 3.

#### 3.4.2. Screening of Key Targets of “Fructus Ligustri Lucidi-Cuscutae Semen” for the Treatment of PCa

We performed PPI network analysis [8] to identify the targets that play a key role in the PPI network. Next, we calculated the values of the network topology characteristic properties of the intersecting PPIs (Figure 3). After three screens were performed, 221 key targets were obtained. The screening parameters included degree centrality (DC), closeness centrality (CC), and betweenness centrality (BC) [9]. The specific screening process and screening parameters are shown in Figure 4. The final core target interaction network is shown in Figure 5.

To more accurately analyse the mechanism of action of “Fructus Ligustri Lucidi-Cuscutae Semen” in the treatment of PCa, it was necessary to identify the intrinsic modules after obtaining the core PPI network. The molecular complex detection algorithm was used to analyse the interactions and obtain the module (Figure 6). The functions of the biological processes in the module are described in Table 2.

### 3.5. Visualization of PCa Pathway Enrichment Analysis for “Fructus Ligustri Lucidi-Cuscutae Semen” Treatment

Two hundred and twenty-one key targets were imported into Metascape for GO function and KEGG pathway enrichment analysis. The results showed that GO function, including BP 1956, CC 66, MF 135, and KEGG enrichment, involved 305 pathways. The top 20 entries of GO and KEGG significance, according to the Log10(*P*) values, were plotted in bubble diagrams using Image GP (http://www.ehbio.com/ImageGP/) (Figure 7). The GO-BP mainly included apoptotic signalling pathways, response to inorganic substances, cellular response to chemical stress, response to oxidative stress, and response to reactive oxygen species; GO-CC mainly involved membrane rafts, membrane microregions, protein kinase complexes, cell cycle protein-dependent protein kinase holoenzyme complex, and serine/threonine protein kinase complex; GO-MF mainly involved transcription factor binding, DNA-binding transcription factor binding, RNA polymerase II-specific DNA-binding transcription factor binding, and protein kinase binding. The KEGG analysis mainly contained pathways in cancer, hepatitis B, AGE-RAGE in diabetic complications, PI3K-Akt, IL-17, and TNF signalling pathway.

### 3.6. Molecular Docking

Molecular docking is a technique that simulates the interaction between ligand small molecules and receptor protein macromolecules. It calculates the binding energy between two counterparts to predict their affinity. A binding energy < 0 indicates that the two molecules bind spontaneously. Moreover, a smaller binding energy results in a more stable conformation. In this study, the target genes, TP53, NTPK1, ESR1, MCM2, and EGFR, with high degree values were selected as receptors. The potentially active components were used as ligands for molecular docking. Most of the potential active ingredients could complete good docking with the target proteins according to the binding energy of receptors and ligands (Table 3). The best docking was between paclitaxel and TP53; quercetin, sesamin, and kaempferol with TP53, and *β*-sitosterol with EGFR and ESR1 also showed good docking (binding energy, ≤ −7 kJ/mol for all). The local structures of molecular docking are shown in Figure 8.

## 4. Discussion

The symptoms of PCa are not obvious in the early stage; difficulty in urination, frequent urination, and erectile dysfunction appear in the middle and late stages of PCa. From a macroscopic perspective, the pathogenesis of PCa is related to factors such as advanced age, genetics, and prostatitis. From a microscopic perspective, genetic gene mutations such as BRCA1/2 and ESR1, activation of signalling pathways such as PI3K-AKT, and expression of the androgen receptor (AR) are potential pathogenic mechanisms leading to the proliferation and migration of PCa cells [6, 10, 11]. Studies have shown that both Fructus Ligustri Lucidi and Cuscutae Semen can enhance body immunity. Moreover, Fructus Ligustri Lucidi can reduce tumour volume and weight, and Cuscutae Semen can inhibit PCa cell proliferation [12–15]. However, the molecular mechanisms underlying these effects need to be further explored. In this study, we used a network pharmacology and molecular docking approach to elucidate the potential mechanisms underlying the beneficial effects of Fructus Ligustri Lucidi and Cuscutae Semen on PCa.

Using database predictions, we determined that Fructus Ligustri Lucidi and Cuscutae Semen affect PCa through multiple active ingredients. The main active ingredients included taxifolin, quercetin, sesamin, kaempferol, and *β*-sitosterol. Both taxifolin and quercetin are flavonoids. Taxifolin inhibits the production of androgens in Leydig cells, inhibits PCa cell growth, and induces PCa cell apoptosis [16]. Quercetin significantly inhibits the proliferation of PC3 androgen nondependent PCa cells and LNCaP cells, thereby suppressing PCa cell survival [17]. Sesamin is a lignan-like plant fibre compound with powerful anticancer properties. *In vivo* studies have found that sesamin inhibits human PCa cell invasion and adhesion, prevents tumour angiogenesis in PCa cells, exerts powerful antioxidant effects, and attenuates oxidative stress [18]. Therefore, it has become a new PCa drug candidate. Kaempferol is one of the most common glycosidic forms of sesamin flavonoids. It acts by upregulating cystatinase-8, -9, and -3 and poly (ADP-ribose) polymerase protein expression to inhibit PCa cell proliferation [19]. Additionally, it has a significant effect on PCa cell transcription, has low toxicity, and increases survival [20]. *β*-Sitosterol is the most abundant phytosterol in the human. It significantly reduces PCa cell growth, induces apoptosis [21], and modulates 17*β*-HSD4 activity [22].

We analysed the PPI network of potential therapeutic PCa targets and screened the more important targets, TP53, NTRK1, ESR1, MCM2, and EGFR, from 221 core targets. Deletion of TP53 contributes to the development of AR nondependent or neuroendocrine tumour phenotypes into PCa [23–25]. Moreover, TP53 mutations play an important role in clinically guiding the precise treatment of primary hormonal PCa. This which may be achieved by TP53 inhibiting PCa development *via* cell cycle progression control, senescence, DNA repair, and cell death. NTRK1 is a receptor tyrosine kinase that is distributed in prostate tissue. It binds to nerve growth factors on the cell membrane and can activate the Ras/MAPK, PI3K, and PLC*γ* signalling pathways to promote cell survival, proliferation, and invasion [26]. Stronger NTRK1 signals indicate higher malignancy in PCa [27]. SR1 is a receptor for oestrogen, which can activate ESR1 to promote normal prostate development and gene expression in prostate disease [28]. Experimental studies have shown that ESR1 may reduce the risk of PCa by stimulating abnormal prostate growth, controlling prostate cell growth, and programming prostate cell death [29]. MCM2 is a protein belonging to the minichromosome maintenance protein complex (MCM) family. Its luminal cell expression serves as a marker of normal epithelium at high risk for PCa [30] and in neuroendocrine PCa (NEPC). During development, the upregulation of SOX2 and EZH2 drives elevated levels of MCM2, which inhibits the proliferation, replication, and metastasis of NEPC cells [31]. EGFR plays a key role in the rapid clonal expansion of progenitor cells derived from cancer stem cells, which is particularly relevant for solid tumours. Basic studies have found that dual intervention with EGFR and HER2 can deplete tumour initiating cells, optimising chemotherapy management, and preventing the progression of desmoplastic resistant PCa cells [32].

In this study, KEGG enrichment analysis was used to explore the main pathways by which Fructus Ligustri Lucidi and Cuscutae Semen treat PCa. We found that they affect the AGE-RAGE, PI3K-Akt, IL-17, and TNF signalling pathways, which have roles in PCa cell apoptosis, migration, and oxidative stress. The AGE-RAGE signalling pathway activates the inflammatory environment and promotes tumour formation and progression by promoting cancer-related processes, such as ECM remodelling, angiogenesis, and metastasis [32]. Additionally, it plays a role in inducing cell proliferation; basic experimental studies have shown [33, 34] that the V structure of RAGE preferentially interacts with AGE on PCa cells. Moreover, AGE induces cell growth and invasion in PCa cells. The PI3K-AKT signalling pathway plays an important role in PCa genesis and is a key crossover point in the therapeutic process. *In vitro* studies have shown that it is involved in the proliferation, apoptosis, migration, and invasion of PCa cells [35]. The mechanisms of this pathway in PCa genesis are multifaceted and include inflammation, cell cycling, and angiogenesis [36]. IL-17 is a key proinflammatory cytokine that promotes the development of PCa and lymph node metastasis [37]. Enhanced PCa glycolytic activity contributes to the formation of a tumour immune microenvironment. Additionally, this signalling pathway plays an important mediating role in the interaction between tumour glycolysis and immune function [38]. TNF signalling plays an important role in the migration and invasion of PCa cells. Androgen deprivation induces TNF signalling. Further, TNF-mediated prosurvival signalling is a major pathway leading to cell survival and treatment resistance [39]. Taken together, these data show that multiple pathways can interact to influence PCa cell activity. PI3K-AKT signalling pathway regulates Rb phosphorylation to enable AGE-RAGE interactions that enhance PCa cell proliferation [40]. Moreover, IL-17F promotes the malignant phenotype of PCa cells by activating the PI3K-AKT signalling pathway, providing a potential therapeutic target for PCa [41].

The molecular docking results revealed that taxifolin, quercetin, sesamin, kaempferol, and TP53 were targets in Fructus Ligustri Lucidi and Cuscutae Semen. *β*-Sitosterol and EGFR targets and ESR1 targets showed effective binding activities; however, their biological functions for treating PCa need to be further validated.

Androgens promote the development and progression of PCa; targeted AR therapy is a current hot topic in PCa. The active components in Fructus Ligustri Lucidi and Cuscutae Semen found in this study have known antiandrogenic effects. Taxifolin inhibits androgen production in Leydig cells, inhibits PCa cell growth, and induces PCa cell apoptosis [16]. Quercetin blocks AR activity and inhibits PCa development [42]. Kaempferol significantly inhibits dihydrotestosterone (DHT) AR activation, while reducing downstream targets of AR and ultimately inhibiting PCa cell proliferation, angiogenesis, and invasion [43].

Target expression in Fructus Ligustri Lucidi and Cuscutae Semen influences AR activity. For example, deletion of the TP53 target expression signature can lead to a diminished response to AR antagonists [44]. mCM2 and EGFR targets can inhibit AR signalling [45, 46]. Moreover, the signalling pathways related to the active ingredients in Fructus Ligustri Lucidi and Cuscutae Semen are closely related to AR. Downregulation of RAGE expression by RNAi inhibits cell proliferation in both androgen-dependent and androgen-independent PCa cells [47]. The PI3K-Akt signalling pathway is AR-dependent [48] and regulates Rb phosphorylation to enable AGE-RAGE interaction, which enhances PCa cell proliferation [49]. Androgen deprivation induces TNF signalling [40]. Therefore, AR expression is positively correlated with PI3K-Akt, AGE-RAGE, and TNF signalling pathways. This indicates that antiandrogen resistance of Fructus Ligustri Lucidi and Cuscutae Semen may be a result of the activity of taxifolin, quercetin, and kaempferol acting on TP53, MCM2, and EGFR targets to inhibit the PI3K-Akt, AGE-RAGE, and TNF signalling pathways. This leads to the inhibition of AR activity for the treatment of PCa. However, few studies have confirmed this hypothesis; therefore, further experimental evidence is needed.

## 5. Conclusion

In this study, a network pharmacology and molecular docking approach was used to identify taxifolin, quercetin, sesamin, kaempferol, and *β*-sitosterol in Fructus Ligustri Lucidi and Cuscutae Semen. Key genes, such as TP53, NTRK1, ESR1, MCM2, and EGFR, were targeted to identify these active components. The results of the KEGG enrichment analysis indicated that Fructus Ligustri Lucidi and Cuscutae Semen may alleviate PCa by regulating AGE-RAGE, PI3K-Akt, IL-17, and TNF signalling pathways. Taken together, these data suggest that Fructus Ligustri Lucidi and Cuscutae Semen may have a multicomponent, multitarget, and multipathway effect on PCa. This study investigates the possible pharmacodynamic basis and mechanism of action of Fructus Ligustri Lucidi and Cuscutae Semen network pharmacology to predict the therapeutic effect of PCa. The molecular docking results also showed that the active molecules of Fructus Ligustri Lucidi and Cuscutae Semen have good binding activity to key target proteins. This study provides a scientific basis for further experimental studies and clinical applications.

## Figures and Tables

**Figure 1:** The “Ligustrum lucidum-Cuscutae Semen” active ingredient-target network map. The hexagon represents the target of the action of the active ingredient; the quadrilateral represents the 13 active ingredients; NZZ represents Fructus Ligustri Lucidi; TSZ represents Cuscutae Semen; and A is the active ingredient shared by Fructus Ligustri Lucidi and Cuscutae Semen.

**Figure 2:** Venn diagrams of drug targets and disease targets.

**Figure 3:** PPI network diagram of the intersection of “Ligustrum lucidum-Cuscutae Semen” and PCa.

**Figure 4:** Screening strategy diagram for key nodes. DC denotes connectedness centrality, CC denotes compactness centrality, and BC denotes betweenness centrality.

**Figure 5:** “Ligustrum lucidum-Cuscutae Semen” core target interaction network.

**Figure 6:** The inner potential module network of the core PPI network of “Ligustrum lucidum-Cuscutae Semen” in the treatment of PCa. (a–e) are the six functional groups with biological assemblage significance.

**Figure 7:** Bubble chart of enrichment bubbles of targets for the treatment of PCa by “Ligustrum lucidum-Cuscutae Semen.” (a) GO-BP analysis; (b) GO-CC analysis; (c) GO-MF analysis; (d) KEGG analysis.

**Figure 8:** Molecular docking results of potential active components and targets for the treatment of PCa in “Ligustrum lucidum-Cuscutae Semen.” (a) stands of taxifolin and TP53; (b) stands of quercetin and TP53; (c) stands of sesamin and TP53; (d) stands of beta-sitosterol and EGFR; (e) stands of kaempferol and TP53; (f) stands of beta-sitosterol and ESR1.

**Table 1:** Potential active ingredient.

ID	Number	Ingredient name	OB/%	DL
NZZ1	MOL004576	Taxifolin	57.84	0.27
NZZ2	MOL005147	Lucidumoside D_qt	54.41	0.47
NZZ3	MOL005190	Eriodictyol	71.79	0.24
NZZ4	MOL005212	Olitoriside_qt	103.23	0.78
NZZ5	MOL000006	Luteolin	36.16	0.25
TSZ1	MOL001558	Sesamin	56.55	0.83
TSZ2	MOL000184	Stigmasterol	39.25	0.76
TSZ3	MOL000354	Isorhamnetin	49.60	0.31
TSZ4	MOL005440	Isofucosterol	43.78	0.76
TSZ5	MOL005944	Matrine	63.77	0.25
A1	MOL000358	Beta-sitosterol	36.91	0.75
A2	MOL000422	Kaempferol	41.88	0.24
A3	MOL000098	Quercetin	46.43	0.28

**Table 2:** “Ligustrum lucidum-Cuscutae Semen” treats PCa core PPI network internal potential module network function description (top 5).

Entry	Function description	Log_10_(*P*)
GO:0097190	Apoptotic signalling pathway	-24.1
GO:0010035	Response to inorganic substance	-22.5
GO:0062197	Cellular response to chemical stress	-21.1
GO:0048545	Response to steroid hormone	-11.9
GO:0071396	Cellular response to lipid	-10.1

**Table 3:** Binding energy of potential active ingredients to target proteins.

Potential active ingredients	Combined energy (kJ/mol)				
	TP53	NTPK1	ESR1	MCM2	EGFR
Taxifolin	-8.94	-4.37	-2.47	-3.54	-4.07
Lucidumoside D_qt	-4.06	-3.48	-2.82	-3.03	-4.11
Eriodictyol	-5.64	-4.56	-4.97	-3.88	-4.01
Olitoriside_qt	-4.06	-3.48	-2.82	-3.03	-4.70
Luteolin	-4.88	-2.74	-2.67	-5.02	-3.45
Sesamin	-7.69	-6.08	-4.86	-4.71	-4.26
Stigmasterol	-5.69	-4.10	-4.86	-3.01	-4.75
Isorhamnetin	-4.60	-4.80	-2.88	-4.21	-3.54
Isofucosterol	-3.60	-4.11	-4.73	-5.26	-3.54
Matrine	-6.22	-5.04	-4.16	-4.49	-4.30
Beta-sitosterol	-4.58	-4.95	-7.07	-3.22	-7.58
Kaempferol	-7.39	-4.52	-4.06	-3.68	-6.01
Quercetin	-8.74	-3.61	-3.10	-2.29	-3.16

## Data Availability

The datasets used during the current study are available from the corresponding author on reasonable request.
